The article "Music’s ability to foster prosocial behavior: a teleofunctionalist perspective" was published in 2025. Journal: Front Psychol.

# Music’s ability to foster prosocial behavior: a teleofunctionalist perspective

**DOI:** 10.3389/fpsyg.2024.1472136

**Published:** 2025-01-22

**Authors:** Jin Hyun Kim

**Affiliations:** Department of Music and Technology, University of the Arts Helsinki, Helsinki, Finland

**Keywords:** affiliative communicative interaction, proper functions of music, teleofunctionalism, protoconversational communication, musical forms of vitality, shared experiences, basic empathy, shared intentionality

## Abstract

Drawing on recent interdisciplinary music research—biologically or developmental psychologically oriented—which conceptualizes music as a communicative toolkit primarily serving affiliative communicative interaction, this paper investigates the question of whether and to what extent music is capable of fostering prosocial behavior within the framework of teleofunctionalism—a philosophical theory of mind. A teleofunctionalist perspective allows us to specify this question as follows: To what extent might a function of establishing affiliative socio-interactional relationships be considered a proper function of music, a concept suggested by philosopher Ruth Millikan? From an ontogenetic perspective, musical activities are considered to be rooted in protoconversational communication in early infancy, characterized as interpersonal coordination without involving propositional understanding. These activities develop into coordinated, non-representational forms of vitality, involving basic empathy, shared intentionality, and forms of understanding allowing for shared experiences. This effect of musical activities—establishing shared experiences—can be considered a proper function of music. A teleofunctional explanation of why musical practices that foster cooperation and prosocial behavior are reproduced is provided by the participants’ positive evaluation of shared experiences structured by musical activities. By discussing a proper function of a musical activity, the author refines her own considerations concerning the minimal necessary conditions of music and musicality that can be conceived in a broader sense.

## 1 Introduction

In examining whether and to what extent music is capable of fostering prosocial behavior, which is regarded by many authors as a possible adaptive function of music (Roederer, 1984; Storr, 1992; McNeill, 1995; Merker, 1999; Mithen, 2006; Dissanayake, 2008: Patel, 2008, 2018; Dunbar, 2012; Morley, 2013; Tarr et al., 2015; Podlipniak, 2016; Harvey, 2017; Savage et al., 2021), it is important to discuss first what we mean by *music*. This paper addresses a topic of basic music research: determining what makes certain artifacts and practices created and performed in a given culture “musical” or “music-like”.^1^ In doing so, this paper ties to very recent interdisciplinary music research suggesting that music is, like language, a communicative toolkit—which, however, unlike language, primarily serves affiliative communicative interaction (Whiteman, 2020; Cross, 2022; Shilton, 2022).

Music cognition researcher Ian Cross claims that musical interaction is comparable to phatic verbal conversation, as both involve behavioral features that can be aligned in form and periodicity (cf. Cross, 2022, p. 4). Taking the similarities of verbal conversation and musical interaction, which Cross points out, into account, speech should not be characterized as exclusively linguistic: As an important function of linguistic interaction is communicating ideas, based on the representational semantics of language, rather than promoting the interactants’ group affiliation (Bühler, 1934; Larson and Segal, 1995; Speaks, 2021), speech that fosters affiliative interaction among speakers might therefore also be assigned to a musical domain. Cultural evolution researcher Dor Shilton takes up Cross’ claim to this end, considering music “part of a greater communicative toolkit [being] interwoven into different communicative registers and rituals” (Shilton, 2022, p. 2), rather than isolated from other forms of communication. For Shilton, music and language in general have different communicative goals: While language has an explicit communicative goal largely extrinsic to linguistic interaction (e.g., conveying representational semantic meaning), music is mainly directed towards “the participants’ rhythmic, gestural and vocal coordination” (Shilton, 2022, p. 3), which is an intrinsic goal (Whiteman, 2020; Shilton, 2022). Although it is possible to achieve this kind of coordination in dyadic interaction—as in the case of speech-based communicative interaction, which can be characterized as musical as discussed above—speech also contributes to linguistic interaction having an extrinsic goal and, accordingly, is primarily embedded in the dialogic context (Haiduk and Fitch, 2022). Music, conceptualized as a communicative interaction, is however capable of an exponential increase in group size, allowing everyone to contribute to that interaction simultaneously (Weinstein et al., 2016; Tarr, 2017; Savage et al., 2021; Shilton, 2022; Dunbar, 2023); this is characterized as the choric context (Haiduk and Fitch, 2022), although musical interaction can also involve turn-taking (Levinson, 2013; Wöllner, 2018; Kim, 2023a), as in antiphony in Western classical music, the relationship between solos and rhythmic sections in Jazz, or the call and response section between the lead singer and chorus—“Coro-pregón”—found in Caribbean musical genres including salsa and rumba.

Shilton claims that such affiliative interactions involve biobehavioral synchrony on a psychological level. “Biobehavioral synchrony” refers to the coordination of biological processes and species-typical behaviors expressed during or immediately after social contact (Atzil et al., 2014; Feldman, 2012a,b, 2017). Indeed, biobehavioral synchrony underlies collective recitation of prayers (Saraei et al., 2024) and serves as a mechanism for turn-taking in speech conversation (Nguyen et al., 2023; Yokozuka et al., 2021) as well as joint music-making (Clayton et al., 2005, 2021; Tarr, 2017; Kim et al., 2019; Savage et al., 2021) and dance (Tarr, 2017). When considering empirical evidence of the relationship between biobehavioral synchrony and human attachments (Feldman, 2017), and of the neural and neurophysiological correlates between behavioral alignment and alignment of some dynamic affective and attitudinal states (Müller and Lindenberger, 2011; Pan et al., 2018; Hoehl et al., 2020; Shehata et al., 2021), it is possible to assume that there would also be a correlation between biobehavioral synchrony and prosocial behavior. Indeed, several empirical studies have provided empirical findings that biobehavioral synchrony increases prosocial behavior (Wiltermuth and Heath, 2009; Cirelli et al., 2014; Rennung and Göritz, 2016; Stupacher et al., 2017; Cirelli, 2018; daSilva and Wood, 2024; for a review in more detail see Tarr et al., 2014). Moreover, some researchers provide evidence that biobehavioral synchrony that occurs in musical contexts influences prosocial behavior opposed to that in non-musical contexts (Kirschner and Tomasello, 2010; Demos et al., 2012), which is supported by evolutionary psychologist Tarr’s claim that music serves as a shared and predictable rhythmic scaffold, facilitating interpersonal synchrony (Tarr, 2017).

Is the status of music as involving biobehavioral synchrony, however, sufficient for claiming that music is capable of fostering prosocial behavior? To address music’s ability to foster prosocial behavior, the question of the extent to which a social function—more precisely: a function of establishing affiliative socio-interactional relationships—might be considered a proper function of music deserves more thorough discussion. Hence, this paper attempts to refine the author’s own considerations concerning the minimal necessary conditions of music and musicality that can be conceived in a broader sense (Kim, 2023a), taking a philosophical perspective within the framework of teleofunctionalism developed by Ruth Millikan, who suggests the concept of proper function.

## 2 Proper functions of music

Against this background suggesting a conceptualization of music as a tool for affiliative communicative interaction, it is possible to investigate the proper functions of music through posing a more specific question: What proper functions does a *musical activity* have? A musical activity refers to an activity in which those phenomena and behaviors that are described as “musical” or “music-like” in a given culture are created or exhibited, for instance, singing, playing an instrument, and dancing. The new question does not overlook musical works, since they are products created by musical activities; but it shifts the research focus to the activities required to produce and interpret those specific forms of communication that differ from forms of communication—such as linguistic communication—having an explicit communicative goal.

For Ruth Millikan, the proper function of an item is not determined by looking to “[its] present properties or dispositions” (Millikan, 1989, p. 289). The proper function is an effect for which the ancestors of such properties or dispositions were selected for (Roloff, 2023). Although Millikan associates proper functions with reproduced items (Millikan, 1984, p. 17), assigning “the survival value of a reproduced type of entity” to the proper function (Millikan, 1995, p. 186), her notion of proper function does not refer to the specific conditions of biological reproduction and selection (Origgi and Sperber, 2000, p. 143); this is evident as she uses the term “biological” in her seminal monograph *Language, Thought, and Other Biological Categories* (1984) metaphorically rather than literally (cf. Millikan, 2002, p. 115). The proper functions of items addressed by Millikan encompasses “the functions of learned behaviors, reasoned behaviors, customs, language devices such as words and syntactic forms, and artifact” (Millikan, 1989, p. 289).

Millikan introduces the two types of proper function: direct and derived. An item *A* has a direct proper function *F* if the following condition is fulfilled: “*A* originated as a ‘reproduction’ […] of some prior item or items that, *due* in part to possession of the properties reproduced, have actually performed *F* in the past, and *A* exists because (causally, historically because) of this or these performances” (Millikan, 1989, p. 288; Millikan, 1993, p. 12). A direct proper function of an item can therefore be determined by “look[ing] to history” (Millikan, 1989, p. 289). When considering her example of the proper function of hearts that consists of pumping blood (Millikan, 1984, p. 17 f.), it becomes evident that the direct proper function of hearts can thus also be attributed to a defective and therefore malfunctioning heart. An item *A* has a derived proper function *F* if the following condition is fulfilled: “*A* originated as the product of some prior device that, given its circumstances, had performance of *F* as proper function, and that, under those circumstances, normally causes *F* to be performed by *means* of producing an item like *A*” (Millikan, 1989, p. 288; Millikan, 1993, p. 12). This type of proper functions is derived from the function of a device that produces different items that may not be reproduced (Millikan, 1993, p. 12 f.), but has causally relevant properties (Origgi and Sperber, 2000, p. 144). The concept of derived proper function allows us to integrate a discussion of the proper functions of the use of a given musical device under a given context, and can therefore be useful when addressing the culture-specific aspects of the functions of particular musical activities, which, however, can be described generally so as to be considered shared by many other musical activities. Consequently, a thorough investigation of the proper functions of a musical activity from the teleofunctionalist point of view needs to pursue an etiological approach.

According to Millikan, a proper function has two features: the normative and the teleological. Teleological terms are evaluative, but normative terms not necessarily so; normative terms are used to “indicate any kind of measure from which actual departures are possible” (Millikan, 2002, p. 116). When taking the normative notion of proper function into account, discussing whether a musical activity has proper functions would involve asking whether there is proper functioning of a musical activity from which actual musical features^2^ can diverge. From the teleological point of view, on the other hand, it should be examined whether the function of musical features explains why there are given musical features and what they are for (cf. Neander, 1991, p. 454).

The musical features in question comprise the duration, timbre, harmony, etc. of a musical unit. From the music theoretical point of view, a musical unit refers to a unit of musical structure—for instance, a beat for a rhythmic structure, a motive for a melodic structure, or a phrase or a section relevant for musical form. A measure for actual musical features may be, for instance, a temporal coordination of various musical units based on the isochronicity of rhythmic-periodic structure. Actual musical features—such as a polyrhythmic structure involving rhythmic patterns with two or more different meters simultaneously (e.g., three against two), or partially including non-isochronous meters (e.g., 9 divided 2 + 2 + 2 + 3), often used in non-Western music styles (Arom, 2004; London, 2012; Polak and London, 2014; Polak, 2022)—can diverge from this measure. A proper function of such musical features would thus be able to explain why there are isochronous beats or other larger rhythmic-periodic units and what they are for.

To have a proper function, an item must come from a set of items that have been reproduced (a direct proper function) or produced by a device that has a proper function (a derived proper function) due to a positive correlation between features and the functions of these features. Millikan defines the notion of proper function as follows, primarily taking the notion of direct proper function into account:

“Where *m* is a member of a reproductively established family *R* and *R* has the reproductively established or Normal character *C*, *m* has the function *F* as a direct proper function iff:

1. Certain ancestors of *m* performed *F*.
2. In part because there existed a direct causal connection between having the character *C* and performance of the function *F* in the case of these ancestors of *m*, *C* correlated positively with *F* over a certain set of items *S* which included these ancestors and other things not having *C*.
3. One among the legitimate explanations that can be given of the fact that *m* exists makes reference to the fact that C correlated positively with *F* over *S*, either directly causing reproduction of *m* or explaining why *R* was proliferated and hence why *m* exists” (Millikan, 1984, p. 28).

To discuss proper functions of music, a musical activity can be put in place of *m*, whose production results from imitation, which is a member of a reproductively established family consisting of musical responses imitating musical calls *R.* Baroque, contrapuntal compositional techniques constituting a thematic relationship between leading and accompanying voices—including canon, invention, and fugue—are paradigmatic examples in which a leading voice is determined as a melodic structure by the sequencing process, i.e., the production of a temporal sequence of similar musical sections at different pitch levels, which is then imitated by a counterpart voice in a time-shifted or pitch-shifted manner, either retaining the key or pitch intervals unchanged or changing the key or pitch intervals. But imitation techniques are often used in compositional techniques for diverse musical styles, and there are also numerous non-Western and more improvisatory forms of musical imitation.

Likewise, a musical event whose production results from temporal and/or pitch-related and/or timbre-related coordination, can be put in place of *m*. In this case, *R* consists of musically coordinated events having shared musical features, whether rhythmic, melodic or timbral.

Temporal coordination in music involves entrainment, “a process whereby [different (modified by the present author)] rhythmic processes interact with [one another (modified by the present author)] in such a way that they adjust towards and eventually ‘lock in’ to a common phase and/or periodicity” (Clayton et al., 2005, p. 2). This is also the case even where polyrhythmic structures involving non-isochronous meters are used. Several empirical studies show that non-isochrony may be integrated into a metrical framework, within which entrainment serves as a process, as opposed to the assumption that a combination of contrasting rhythmic patterns would not foster entrainment (Yoshida et al., 2002; Polak, 2010; Doffman, 2013; Polak et al., 2016).

A well-known example of pitch-related coordination is collectively singing a birthday song. Even if everyone starts at different pitches, the collective usually ends with nearly the same pitches. Moreover, the discrete pitch features of music, as opposed to the non-discrete pitch in speech (Zatorre and Baum, 2012; Haiduk and Fitch, 2022), serve as the foundation for harmony-based coordination, which I therefore regard as subordinate to pitch-related coordination.

Timbre-related coordination plays a significant role in the timbre-related micro-sonic structures of electroacoustic music, timbre melody, spectral music and overtone singing. Studies on timbre (for an overview, see McAdams and Giordano, 2016) show that dynamic sound properties involving tension and release can also be shaped by dimensions of timbre. Additionally, matching the timbral properties of singers is crucial for a singing ensemble, and aficionados often value the timbre of a singer’s voice when selecting their favorite performers. Consequently, timbre-related coordination is regarded as a relevant process involved in singing with co-singers or listening to a song. When taking into account the well-known fact that temporal pitch-related and/or timbre-related coordination also occurs in speech conversation, specifically focusing on its phatic function (Cross, 2022), it is plausible to suggest that speech should not be characterized as exclusively linguistic and can rather be assigned to a musical domain, as discussed in the introduction.

Such features of a musical activity—isochronous beats, larger rhythmic-periodic units, call and response patterns, and shared rhythm, pitch or timbre—do not represent any state of affairs, and therefore would never be evaluated as successfully fulfilling conditions for a sign that is representationally mapped to some such state. Under which conditions then can a musical activity be evaluated as successful? Conditions under which the mechanisms of producing a musical activity and the mechanisms of interpreting that activity are both selected, based on the producers’ and interpreters’ experiences, and whose structures are mapped to those of musical activity, should be involved. A proper function of such a musical activity would then consist in its effect—which is to establish shared experiences—rather than its purpose.

Most known musical activities throughout history and in various cultural contexts are joint activities, meaning that more than one individual contributes to the activity (Merriam, 1964; Feld, 1982; Seeger, 2004; Turino, 2008; Savage et al., 2015). A musical activity can therefore be considered an activity of inter-individual cooperation, constituting a unity of participants to be understood as a group. Even musical activities that can be performed by a single individual—“solo” in current musical practices—do not serve as a counter example, in that (1) they can be shaped by more than one individual together in principle, (2) the main features of those activities are the same as those cases where further individuals undertake accompanying roles, and (3) the intergenerational transmission of solo repertoire often occurs during active listening (Stubington, 2007; Curran and Yeoh, 2021).

Although there are highly organized joint musical activities, in which the roles of all participants are defined in advance within the framework of a group—for instance, an orchestra or a choir—many joint musical activities, including free improvisation, work songs, and live coding, are based not on a social norm, but rather on a loose cooperation among participants (cf. Kim et al., 2019, p. 9). In such a joint musical activity, musical features being shaped by participants together unfold based on their interpretations of those features, on a moment-to-moment basis until that musical activity is completed. Hence, the production mechanisms are interwoven with the interpretation mechanisms. On the other hand, a series of joint musical activities taking place, especially in ritual contexts, allow interpreters to take part in those activities as co-shapers. In such cases, interpreters serve as producers at the same time; this can result in joint musical activities based on inter-group cooperation, which goes beyond inter-individual cooperation within a group. When considering those cases where producing a joint musical activity is guided by its interpretation and vice versa, it is plausible that there are commonalities between the production mechanisms and interpretation mechanisms underlying a joint musical activity.

Moreover, recent music cognition research suggests that, even in cases where interpreting a musical activity is decoupled from its production—for instance, analyzing Western music in the common practice period from the music theoretical perspective—the interpretation mechanisms are akin to the production mechanisms, such that covert or overt behaviors imitating actions performed by producers underlie certain processes of interpretation (Godøy, 2001, 2010; Cox, 2011, 2016). Those mechanisms are characterized by cognitive music theorist Arnie Cox as motor mimetic imagery and motor mimetic action.

Rather than motor imagery that is considered a representation of motor behaviors involved in specific actions performed by producers (Kim, 2023b), the present author suggests that kinesthetic imagery should be considered a common mechanism of both producing and interpreting a musical activity, regardless of whether the processes of production and interpretation are interwoven with or decoupled from each other. Kinesthetic imagery can be understood as (quasi-)perceptual conscious experience related to dynamic self-movement, which is accessible to phenomenal consciousness (Kim, 2023b, p. 61). A music philosophical concept of re-enactment (*Nachvollzug*) suggested by philosopher Vogel (2007) supports the involvement of motor mimetic action and kinesthetic imagery. He claims that interpreting a musical activity involves a process of understanding that allows for shared experiences, which may occur covertly—involving kinesthetic imagery according to Kim (2023b)—or overtly in terms of a re-enactment of musical features in an intramedial or intermedial way (cf. Vogel, 2007). To give examples for the latter, it is possible that melodic features of an instrumental musical piece are overtly re-enacted either by the interpreter’s singing vocal melodic contours (in an intramedial way) or through their hand gestures (in an intermedial way).

Such mechanisms of interpreting a musical activity considered as shared with the production mechanisms, which have been addressed in recent music cognition research and music philosophy, as discussed above and by further scholars (Godøy, 2001, 2010; Leman et al., 2009; Overy and Molnar-Szakacs, 2009; Cochrane, 2010; Cox, 2011, 2016; Krueger, 2013; Kim, 2013, 2023b; Vogel, 2007), support the view that establishing shared experiences can be conceived of as the effect of a musical activity that is its proper function. This view can, however, be further examined by looking to history in which joint musical activities leading to shared experiences have been reproduced; an etiological view is necessary to determine a proper function of music. From an ontogenetic perspective, the protoconversational communication that takes place in infant-caregiver interaction is considered a basis for both music and language (Trevarthen, 2002; Malloch and Trevarthen, 2009; Van Puyvelde et al., 2010, 2013). Hence, the next section devotes its discussion to the question of the extent to which music is originated from protoconversational communication.

## 3 From protoconversational communication to joint musical activities?

According to infancy researcher Colwyn Trevarthen, protoconversational communication is characterized as interpersonal coordination involving behaviors in sync or in tune with one another, as well as qualitatively attuned behaviors, providing shared rhythmic foundation for periodic matching and shared intonational foundation for prosodic matching and melodic adjustment (Trevarthen, 1999). The co-constructing behaviors of caregiver and infant during their interaction result in a characteristic dynamic Gestalt, which Stern calls “vitality form” (Stern, 2010). This term refers to the form of a living being’s behavior involved in overt actions and covert processes, or of the arts consisting of movement, time, force, space, and directionality, which is relationally constituted through interaction with the world and others (Stern, 2010, pp. 5 f.). Forms of vitality that can be manifested in physical behaviors are related to the way in which those behaviors are exhibited rather than the content of those behaviors, e.g., other’s emotional states. In cases where a behavior that serves as a sign expressing one’s representational mental states exhibits forms of vitality, those forms of vitality could contribute to an understanding of representational content of that sign.

But there are also cases where forms of vitality come into the foreground because: (1) there are no representational mental states behind a behavior, or (2) the interpreters of vitality forms do not have the capacity of mind-reading. Interestingly, Stern points to “content free vitality forms” (Stern, 2009, p. 315), which are paradigmatically observed in interactive behavior of a 2–3-month-old infant exhibited as a response to their caregiver’s body movements and voices (cf. Stern, 1985, p. 143). The capacity of mind-reading is generally observed in the later stages of childhood, i.e., at 7–18 months (cf. Buttelmann et al., 2009; Carruthers, 2013). Hence, protoconversational communication in early infancy involves non-representational forms of vitality. This means that infant and caregiver do not feel the same emotion during their protoconversational communication, but shape “coordinated non-representational forms of vitality” (Kim, 2023a). Trevarthen calls the innate capacity of producing forms of vitality and appreciating other’s forms of vitality “communicative musicality” (Malloch and Trevarthen, 2009, 2018).

The term “communicative musicality” is debateable, as the meaning of “musicality” presupposes an understanding of what music is or does. Likewise, the concept of musicality supported in current bio-musicological research (Fitch, 2015; Honing et al., 2015; Honing, 2018; Savage et al., 2021)—as a natural, spontaneously developing trait based on and constrained by our cognitive abilities and their underlying biology, as opposed to music that is conceived as a social and cultural construct based on that very musicality—is not driven by the concept of music.^3^ Unlike protoconversational communication in early infancy, musical activities involve shared intentionality (Gilbert, 1990; Bratman, 1992; Searle, 1995; Tuomela, 2013; Tomasello, 2014)—either collective intentionality (Tuomela, 2013; Tomasello, 2014), or at least we-intentions (Searle, 1990, 1995)—to create musical units that are considered meaningful in a given culture by shaping sounds and bodily movements. We-intentions, which are weaker than collective intentionality, are not supradindividual intentions: Rather, the I-mode intentions of each interactant are expressed with reference to others while performing a cooperative activity (Searle, 1990, p. 406 f.). Collective intentionality is a strong kind of shared intentionality, involving a “we-mode” of each interactant (Tuomela, 2013), who represents the group through a specifically defined role in the group (Tuomela, 2013, p. 15; cf. Kim et al., 2019, p. 8).

As a result, it is difficult to assign musicality to protoconversational communication that does not necessarily involve we-intentions. Early infant-caregiver interaction is based instead on inter-individual behavior leading to social interaction, without any shared intentionality (Reddy, 2008; Feldman et al., 2009; Fantasia et al., 2014; León, 2021; for a more detailed discussion see Kim et al., 2019, p. 7) This kind of behavior consists of each interactant’s own activity in a causal relation to a shared social context that affords or constrains each interactant’s selection of their behavior, as well as the perception of their own and others’ behavior. Behavior that emerges in the course of reciprocation is not considered to be derived from shared intentionality (Kim et al., 2019; Moll et al., 2021).

On the other hand, protoconversational communication aiming at interpersonal coordination—rather than at conveying representational meanings—during behavior-based dyadic interaction presupposes an innate ability of human beings which is also necessary for musical activities: namely, hetero-directed competence. In current empathy research, empathy based on the inner activity of movement is called “basic empathy” (Stueber, 2006; Gallagher, 2012). Unlike the Simulation Theory of Theory of Mind, which discusses empathy as if it is based on the simulation of other’s mental states (Goldman, 2006), the concept of basic empathy can be conceived of as being based on hetero-directed competence related to others, but not necessarily to other’s representational mental states. Although empathy has been assiduously discussed as an intersubjective relation in current philosophy of mind, social neuroscience, and related research areas, this notion of basic empathy should be related to the original concept of empathy suggested by Robert Vischer and further developed by Theodor Lipps at the end of 19th and beginning of 20th century. This concept was about a relation with objects (Currie, 2011), especially as a process underlying aesthetic experience—including that of music. Basic empathy can be considered one of the primary mechanisms of producing and interpreting both protoconversational communication and joint musical activities.

From an ontogenetic perspective, the caregiver’s affective attunement has a function of sensitization (Marraffa and Meini, 2019). The infant becomes sensitive to the set of physiological and proprioceptive cues, which are not necessarily representational, while their behaviors exhibiting forms of vitality affect the caregiver’s responses; the intimate skills of an affectively attuned caregiver helps the infant at later stages of infancy manage and discover more refined forms of vitality which can be considered meaningful in a given culture, although, unlike a linguistic-semantic unit, those units rarely bear any representational meanings (Kim, 2023a). Nonpropositional regulations of internally generated motives and self-awareness shared intimately between human beings could develop in this way, leading to skills in the formation of musically meaningful units that can be called musical forms of vitality (Kim, 2013), involving shared intentionality.

Musical forms of vitality can be analyzed in terms of intra-musical relations such as repetition or imitation of a musical element through another musical element; yet shaping such forms is based on a coordinated process of joint musical activities, so that seemingly intra-musical relations can be expressed in terms of social relations. Musical others are not only (co)musicians, composers or virtual persons, but also musical forms of vitality providing a kind of social biofeedback (Gergely and Watson, 1996). An implicit and immediate process related to musical others is the basic empathy discussed above. Basic empathy that underlies a process of sharing and co-shaping a musical activity is directed towards musical forms of vitality, which structure shared experiences. Establishing shared experiences through musical activities relies not only on an ability for interpersonal coordination, but also on an ability for understanding musical forms of vitality as meaningful in a given culture, based on shared intentionality. Accordingly, minimal necessary conditions of music and musicality that can be conceived in a broader sense might be refined by more specifically discussing a proper function of music.

## 4 Discussion

Considering protoconversational communication as a basis for musical activities allows scholars to discuss the social functions of music from a perspective on social cognition, which does not consist in observing others and reading their mental states but in participating in interaction. This shift from an isolationist to an interactive perspective on social cognition (Becchio et al., 2010; Schilbach et al., 2013) accordingly provides a pragmatic framework for discussing a proper function of music. By asking what proper functions a *musical activity* has, this paper, comparable to Small’s concept of musicking (Small, 1998), attempts to take a pragmatic dimension of the practices that can be described with emic expressions that are identified as synonymous with “music” or, from a musicological perspective, as “music” or “music-like” for granted. It is concerned with an attempt to determine the minimal necessary conditions of music and musicality that can be conceived in a broader sense.

Musical units that can be viewed as units of musical activities that coordinate with one another (cf. Levinson, 2013) embody forms of social behavior relating to the world, which can be characterized as forms of vitality (cf. Kim, 2013, 2023a). A relation of behavior to the world implies a process of understanding, since understanding the world singles out relevant aspects of the world. Joint musical activities, involving shared intentionality, are produced and interpreted by human beings whose nature consists in understanding the world. It is therefore necessary to highlight a hermeneutic dimension—in addition to a pragmatic dimension—to refine the minimal necessary conditions of music and musicality. For this, however, the established theory of metarepresentational understanding (Detel, 2011, 2014), focusing on assessing representational mental states, signs, and actions, is not applicable. Rather, the question of the relationship between the human capacity for understanding and the basic ability for coordination and cooperation is of particular importance for a novel hermeneutic approach, which would be appropriate for investigating non-propositional and non-metarepresentational forms of understanding such as musical understanding. In this respect, it is plausible that a form of communication between infant and caregiver that does not involve propositional understanding is considered a basis for music.

As recent music cognition research and music philosophy suggest that the mechanisms of interpreting a musical activity are shared with the production mechanisms (see the section “Proper functions of music”), both *interpretanda* and the mechanisms of interpreting musical activities can be considered to exhibit shared structures. The interpreter’s experiences are co-shaped while engaging in a musical activity being shaped through interaction with others. Since a musical activity develops into coordinated, non-representational forms of vitality, it can be assumed that the interpreter’s experiences have structures that are mapped to those of musical activity, namely coordinated, non-representational forms of vitality. As a result, it can be claimed that forms of understanding that are involved in musical activities allow for shared experiences. A positive evaluation of shared experiences that are structured while engaging in musical activities explains why musical practices that foster cooperation and prosocial behavior are reproduced.

Against this background, minimal necessary conditions of music that can be conceived in a broader sense (Kim, 2023a, p. 66 f.) are refined as follows: communicative practices that can be described as “musical” are characterized as affiliative communicative interaction consisting of sounds and/or body movements; during these practices, coordinated, non-representational forms of vitality are (co)shaped, involving basic empathy, we-intentions or collective intentionality, and forms of understanding that allow interactants to share structured experiences. These practices, although they do not bear any representational semantics, are considered meaningful in that act of understanding occurring in terms of interactive participation and embodied re-enactment.^4^ Consequently, musicality can be defined in a broader sense as an ability to initiate and take part in affiliative communicative interaction consisting of sounds and/or body movements, involving (co)shaping coordinated, non-representational forms of vitality, and the capacity for basic empathy, shared intentionality (at least, we-intentions), and experience-structuring nonverbal understanding in form of interactive participation and embodied re-enactment.

## Footnotes

^1^For this characterization of basic music research, I fall in with the view of ethnomusicologist and social anthropologist John Blacking (Blacking, 1995, p. 224) that “… every known human society has what trained musicologists would recognise as ‘music’” although “there are some that have no word for music or whose concept of music has a significance quite different from that generally associated with the word ‘music’”.

^2^In this paper, the term “feature” is used instead of the biological term “trait” to extend the discussion about proper functions of music to the cultural conditions under which musical activities are produced and interpreted.

^3^Once minimal necessary conditions of music are determined, a proper definition of musicality can be suggested; this is one of objectives of this paper and will be presented in the section “discussion”.

^4^This concept of music encompasses dance, as suggested by Tarr with her concept of musicking including music-making and dance (Tarr, 2017), and is therefore conceived in a broader sense than the Eurocentric concept frequently encountered. The implications of this concept, however, deserve more extensive discussion in a separate article, incorporating many examples of various non-European musical practices.
